This article has been retracted.

# The Relevance of Interventional Time and Clinical Outcomes in Patients with NSTEMI Based on the GRACE Score

**DOI:** 10.1155/2022/7614619

**Published:** 2022-04-29

**Authors:** Ji-Xiang Wang, Jing Gao, Jian-Yong Xiao, Ming-Dong Gao, Nan Zhang, Peng-Ju Lu, Yin Liu

**Affiliations:** ^1^Cardiology Institute, Tianjin Chest Hospital, Tianjin 300222, China; ^2^Institute of Cardiovascular Diseases, Tianjin Chest Hospital, Tianjin 300222, China

## Abstract

**Objective:**

To investigate the relevance between interventional time and clinical outcomes in non-ST-elevation myocardial infarction (NSTEMI) patients of different risk stratifications, which were divided into different groups according to GRACE scores and the time from admission to percutaneous coronary intervention (PCI).

**Method:**

Patients were grouped according to the GRACE score and the time from admission to intervention therapy. The Cox multivariate risk regression model was used to analyze the correlation between the GRACE score and the time from admission to intervention therapy with major adverse cardiovascular events (MACEs). Cox interactive item regression was also used to investigate the correlation between the time of intervention therapy and GRACE risk stratification with clinical outcomes and to evaluate the efficacy of intervention therapy in different risk stratifications of patients with NSTEMI.

**Results:**

Interactive item Cox regression analysis and subgroup analysis show that high-risk NSTEMI patients with a GRACE score > 140 points and the time from admission to intervention < 24 h (*p* = 0.0004) and 24–72 h (*p* = 0.0143) have interactive effects on the impact of the MACE event with the reference of intervention time > 72 h and GRACE score < 108 points. The time from admission to intervention < 24 h is an independent protective factor for the occurrence of MACE events (HR = 0.166, 95% CI 0.052-0.532, *p* = 0.0025). Middle-risk patients with NSTEMI with a GRACE score of 109–140 points and the time from admission to intervention < 24 h (*p* = 0.0370) and 24–72 h (*p* = 0.0471) have an interactive effect on the impact of MACE. The time from admission to intervention > 72 h is an independent protective factor for the occurrence of MACE (HR = 0.201, 95% CI 0.045-0.897, *p* = 0.0355).

**Conclusion:**

The time from admission to intervention < 24 h could effectively reduce the risk of MACE events within 1 year in high-risk patients with NSTEMI (GRACE score > 140 points); the time from admission to intervention > 72 h can reduce the risk of MACE events within 1 year in low-risk patients with NSTEMI (GRACE score ≤ 108 points).

## 1. Introduction

Acute myocardial infarction (AMI) consists of ST-elevation myocardial infarction (STEMI) and non-ST-elevation myocardial infarction (NSTEMI) via electrocardiography (ECG) diagnosis. In the past 20 years, the proportion of NSTEMI has increased [1] among patients with acute coronary syndromes (ACSs), accounting for 60–75% of patients with AMI [2]. NSTEMI is a common type of coronary heart disease with complicated treatment and poor prognosis [3, 4]. Studies have shown that patients with NSTEMI have a better short-term prognosis and a poorer long-term prognosis [5, 6]. Compared with STEMI, people generally pay less attention to NSTEMI, which poses a challenge to the treatment. Although the mortality rate of patients with NSTEMI has decreased slightly after the universal usage of interventional therapy [7–9], the risk of long-term death still remains a challenge [10, 11]. In recent years, most studies have been conducted in patients with NSTE-ACS to guide the better timing of interventional therapy for patients with NSTEMI based on risk scores. The GRACE study explored independent risk factors affecting the prognosis of patients with ACS (including STEMI, NSTEMI, and UA) [12]; however, these data were not specifically targeting patients with NSTEMI and failed to include Chinese patients. At present, there are few reports on the interventional treatment strategies of patients with NSTEMI worldwide. Therefore, to investigate the relationship between GRACE scores of patients with NSTEMI and the timing of different interventional treatments and clinical outcomes, we performed this study based on the first single-center large sample NSTEMI cohort in China.

## 2. Methods

### 2.1. Study Population

This is a single-center cohort study and included 1357 patients with NSTEMI admitted to the Tianjin Chest Hospital from January 2018 to December 2021.

Inclusion criteria are as follows: (1) aged over 18 years; (2) met the diagnostic criteria for NSTEMI, troponin exceeding the 99% upper limit of reference value, and accompanied by one of the following symptoms: (i) the ST segment was depressed or the T wave was inverted in ECG and (ii) chest pain persists which exceeded 30 minutes; (3) the onset time being less than 30 days; and (4) not participating in other researches in the same period.

Exclusion criteria are as follows: (1) chest pain caused by noncardiac causes, such as aortic dissection, pulmonary embolism, etc.; (2) myocardial infarction with persistent ST-segment elevation during diagnosis and treatment; and (3) not suitable for antiplatelet treatment due to active hemorrhage, severe thrombocytopenia, and so on. This study was approved by the ethics committee of Tianjin Chest Hospital (no. CH2017112002).

### 2.2. Data Collection

The clinical data of patients were obtained by the medical records. The collected data included the patient's basic conditions (age, gender, smoking history, etc.), past history, physical examination, laboratory tests, cardiac color Doppler ultrasound, coronary angiography, and interventional treatment. Laboratory examinations, color Doppler ultrasound, and physical examination were obtained from the first evaluation after admission. Peripheral venous blood samples were collected after admission and analyzed shortly after sampling.

### 2.3. Medical Treatment

According to the timing of coronary angiography and revascularization strategy, PCI, coronary artery bypass surgery, and drug treatment were performed by experienced surgeons and, if necessary, determined by cardiologists and cardiac surgeons together. All patients were divided into 3 subgroups: <24 h, 24–72 h, and >72 h by the time from admission to intervention. According to the GRACE score, there were 3 subgroups: ≤108 points, 109–140 points, and >140 points.

### 2.4. Study Definitions and Clinical Follow-Up

All patients were followed up by electronic medical records, outpatient service or telephone follow-up during the one month, three months, six months, and twelve months after discharge. The follow-up time duration was 1 year, and major adverse cardiovascular events (MACEs) were recorded, which included all-cause death, recurrence of nonfatal AMI, severe heart failure (HF) requiring hospitalization, target lesion revascularization (TLR), and stroke. TLR was defined as a revascularization (PCI or CABG) of the target lesion due to ischemic symptoms or objective evidence, and the stenosis of the target lesion is >50%. Outcomes were divided into primary end point—all-cause death—and secondary end point—MACE events. If the patient showed more than one clinical event, only the first event would prevail and the follow-up would be stopped. According to the occurrence of MACE events, there were the MACE group and non-MACE group.

### 2.5. Statistical Methods

All statistical analyses were performed by SPSS software, version 22.0. According to the GRACE score, the subjects were divided into the low-risk group (≤108 points), medium-risk group (109–140 points), and high-risk group (>140 points). For continuous variables, differences between groups were evaluated with the ANOVA test. Data were presented as mean ± SD. For discrete variables, differences between groups were analyzed with the *χ*^2^ test and were expressed as frequency (percentage). The Kaplan-Meier survival curve was used to analyze the cumulative event rate. Cox-proportional hazard models were used to assess the risk factors of MACE events. Taking MACE events as the dependent variable, the time from admission to intervention (<24 h, 24–72 h, and >72 h), GRACE score (≤108 points, 109–140 points, and>140 points), and the parameters with statistical difference between the occurrence and nonoccurrence of MACE were introduced as covariates into the Cox regression equation. Single-factor regression analysis was performed firstly, and then, the significant variables were included in the multivariate Cox regression analysis to assess the hazard ratio (HR) and 95% confidence interval (CI). The influence of the GRACE score and intervention time on MACE events was found based on the Cox interactive regression analysis. For all analysis, *p* < 0.05 was considered statistically significant.

## 3. Results

### 3.1. Baseline Data of NSTEMI Queue

The average age of 1357 patients with NSTEMI was 64.7 years, and the average length of hospitalization was 6.76 ± 3.87 days. The proportion of male patients was 69.6%. The numbers of patients with GRACE scores in low-, medium-, and high-risk groups were 413 cases (≤108 points, 30.43%), 506 cases (109–140 points, 37.29%), and 438 cases (>140 points, 32.28%), respectively. The baseline characteristics comparison between groups are shown in Table 1. The number of patients who received conservative treatment, interventional treatments, and CABG surgical treatment after admission were 472 (34.78%), 770 (56.74%), and 115 (8.47%). Among them, the majority population were at middle or low risk (*p* ≤ 0.001) and no statistical significance was found between the GRACE groups with CABG treatment. There were 91 patients (6.71%) whose time from admission to intervention was <24 h, 110 patients (8.11%) whose was 24–72 h, and 509 patients (37.51%) whose was >72 h. No significance was found between GRACE groups in patients who received interventional therapy within 24 h (*p* = 0.375).

### 3.2. Clinical Outcomes

Among the 1357 patients with NSTEMI, 1264 cases were followed up for one year but 93 cases were lost (6.85%). A total of 209 cases (16.53%) with MACE events were followed up within 1 year, including 57 cases (4.51%) of all-cause death, 29 cases (2.29%) of relapsed nonfatal AMI, 58 cases (4.59%) of TLR, 78 cases of severe HF (6.17%), and 6 cases of stroke (0.47%) **(**Figure 1**)**.

A total of 658 patients received interventional therapy and completed the follow-up within 1 year. The incidence rates of MACE in the low-risk group (239 cases) who received interventional therapy within 24 h (26 cases), 24–72 h (42 cases), and >72 h (171 cases) were 11.54%, 9.3%, and 2.35% (*p* = 0.031), respectively. The incidence rates of patients in the middle-risk group (265 cases) received interventional therapy within 24 h (27 cases), 24–72 h (39 cases), and >72 h (199 cases) were 3.70%, 2.56%, and 10.55% (*p* = 0.168), respectively. The incidence rates of patients in the high-risk group (154 cases) received interventional therapy within 24 h (31 cases), 24–72 h (20 cases), and >72 h (103 cases) were 9.68%, 15%, and 45.63% (*p* = 0.0002), respectively (Table 2**).**

### 3.3. Multivariate Cox-Proportional Regression Analysis for MACE Events

The results of multivariate COX regression analysis showed that after adjustment, the time from admission to intervention therapy > 72 h (with time < 24 hours as reference) (HR = 4.99, 95% CI 2.25-11.08, *p* < 0.0001), age (HR = 1.035, 95% CI: 1.013-1.058, *p* = 0.002), GRACE score > 140 points (with GRACE score ≤ 108 as reference) (HR = 1.477, 95% CI: 1.765-2.750, *p* < 0.0001), Hs-cTnT (HR = 1.15, 95% CI: 1.04-1.27, *p* = 0.0066), and ≥1 vessel occlusion (HR = 1.54, 95% CI: 1.04-2.27, *p* = 0.0301) are independent risk factors for MACE **(**Table 3**)**.

### 3.4. GRACE Risk Stratification and Regression Analysis and Subgroup Analysis of Intervention Time

1. The results of multivariate COX regression analysis showed that the time from admission to intervention and the GRACE score were independent risk factors for the occurrence of MACE events. To explore the impact of the interaction between the two on the MACE events, interaction terms were added into the regression model. After interactive item regression analysis, we found that the GRACE score > 140 points and the time from admission to intervention < 24 h (*p* = 0.0004) and 24–72 h (*p* = 0.0143); the GRACE score of 109–140 points and the time from admission to intervention < 24 h (*p* = 0.0370) and 24–72 h (*p* = 0.0471) had interactive effect on the MACE event with the reference of intervention time > 72 h and GRACE score < 108 points
2. After subgroup analysis under different GRACE risk stratifications, the effect of intervention time on MACE events showed that for high-risk patients (GRACE score > 140 points), intervention time < 24 h is a protective factor for MACE (HR = 0.166, 95% CI: 0.052-0.532, *p* = 0.0025) (compared with intervention time > 72 h); for low-risk patients (GRACE score ≤ 108 points), intervention time > 72 h is a protective factor for MACE (HR = 0.201, 95% CI: 0.045-0.897, *p* = 0.0355) (compared with intervention time < 24 h) (Figures 2 and 3)

## 4. Discussion

The principal findings of our study are as follows: among patients with NSTEMI, low-risk population with a GRACE score > 140 points should be able to receive intervention therapy within 24 h after admission and low-risk patients with a GRACE score ≤ 108 points should be treated within 72 h. Then, the risk of MACE within 1 year would be reduced effectively. For the middle-risk population with a GRACE score of 109–140 points, the time from admission to intervention treatment would not affect the long-term prognosis.

In this study, the average age of the patients with NSTEMI was 64.7 years, of which 69.6% were male, and these were similar to the total NSTEMI population based on the studies of TIMI [13]. The statistics of this study showed that the NSTEMI patient's 1-year mortality rate is 4.51%, which is lower than the 6.44% of the domestic CAMI study [12]. Compared with foreign statistics, the 1-year mortality rate was slightly higher than the 4.3% of the TIMI-NSTEMI-RCT cohort, lower than 14.3% of the Swedish “SWEDEHEART” study in 2014 [14], the 18.7% of the United States in 2005 [5], and the 12.40% of the French TAO study [15]. The incidence of MACE within 1 year was also low at 16.53%.

It is still controversial of the timing of NSTEMI intervention. The 602 patients with NSTEMI were included in “LIPSIA-NSTEMI” randomized controlled trial, and they were randomly divided into a coronary angiography group (201 cases) within 2 h, a coronary angiography group (200 cases) within 10–48 h, and selective coronary angiography group (201 cases) [16]. This study found that there was no difference in the composite end-point incidence of all-cause death, refractory angina, and rehospitalization at 6 months (26.0% vs 26.5% vs 24.5%; *p* = 0.91). The “VERDICT” trial with different conclusions included 2147 NSTE-ACS patients with new ischemic manifestations or elevated troponin in ECG, which were randomly divided into an intervention group within 12 hand 48–72 h. There was no significant difference between the two groups of cardiovascular events at a follow-up of 4.3 years (HR = 0.92, 95% CI: 0.78–1.08), but intervention strategies within 12 h in high-risk populations with a GRACE score > 140 points could improve long-term prognosis (*p* = 0.023) [17]. The difference between the conclusions of the two studies is the distinction of high-risk population. There are 5 independent risk factors for MACE events within 1 year in patients with NSTEMI: age, GRACE score > 140 points, the time from admission to intervention > 72 h, Hs-cTnT, and ≥1 vessel occlusion. Among them, GRACE > 140 points, time from admission to intervention > 72 h, and vascular occlusion are the strongest predictors of MACE. Meta-analysis studies have shown that criminal vascular occlusion is a risk factor for increased risk of MACE in patients with NSTEMI (1.32, 95% CI: 1.11-1.56, *p* = 0.001) [18]. Therefore, how to use risk stratification to identify these high-risk NSTEMI populations is essential for early intervention and improved prognosis. Early revascularization treatment strategy based on risk scores is more conducive to reduce cardiovascular events, which is the focus of the current research.

The clinical guidelines used to evaluate the risk of patients with NSTEMI mainly include the TIMI score, PURSUIT score, and GRACE score. Among them, the GRACE score is superior to other methods in predicting the risk of cardiovascular events during hospitalization and 6 months and 1 year after discharge, which is a classical scoring system for evaluating the short-term and long-term prognoses [19, 20]. European and American guidelines also recommend the use of GRACE for risk assessment and treatment [21, 22]. However, according to the risk stratification of intervention strategies in the guidelines, NSTEMI can only be divided into very high-risk groups (intervention treatment within 2 h after admission) or high-risk groups (intervention treatment within 24 h after admission). The main difference between the two groups is the evaluation of the patient's clinical situation, such as hemodynamic instability and recurrent chest pain which is difficult to control with medical treatment. Therefore, GRACE risk stratification, as an objective and classic scoring system, has a unique clinical value for NSTEMI intervention timing. After an analysis of patients with NSTEMI based on GRACE risk stratification, we found that for high-risk patients with NSTEMI with a GRACE score > 140 points, the time from admission to intervention < 24 h is a risk for the occurrence of MACE (HR = 0.166, 95% CI 0.052-0.532, *p* = 0.0025). However, for low-risk patients with NSTEMI with a GRACE score ≤ 108 points, the time from admission to intervention < 24 h is a risk factor for the occurrence of MACE within 1 year (HR = 4.984, 95% CI 1.115-22.278, *p* = 0.0355).

Some large studies have confirmed that early intervention therapy can improve the prognosis of high-risk patients. The TIMACS study included 3031 NSTE-ACS patients with a 6-month follow-up. For high-risk NSTE-ACS patients with GRACE > 140 points, early intervention could prevent the risk of end-point events from 35% compared with delayed intervention therapy [23]. The VERDICT study also concluded our study and the TIMACS study: early PCI can benefit patients with NSTE-ACS with a GRACE score > 140 points (HR = 0.81, 95% CI: 0.67-1.00) [17]. On the contrary, delayed treatment will increase the risk of patients. Another study also showed that delayed intervention treatment significantly increased the 30-day risk period and 1-year follow-up mortality and nonfatal AMI incidence.

Patients with ACS are recommended to receive coronary angiography or interventional therapy according to the lesion condition as soon as possible [24]. Our study also reached a similar conclusion: for patients with NSTEMI, the time from admission to intervention > 72 h (HR = 4.99, 95% CI: 2.25-11.08) is a risk factor for MACE within 1 year.

The TAO study provided sufficient evidence-based medicine on the issue of the best intervention time for high-risk NSTEMI populations. It was a clinical study including 4071 high-risk patients with NSTEMI with a GRACE score of >140 points and was to evaluate the impact of interventional strategies of the early period (within 12 h), mid-term period (12–24 h), and delayed period (over 24 h) on prognosis [14]. The follow-up period was 6 months, and the main endpoints were death and relapsed AMI. Finally, we found that very early PCI within 12 h could benefit patients with high-risk NSTEMI (OR = 0.71 95% CI: 0.55-0.91). However, mid-term PCI (OR = 0.96, 95% CI: 0.75-1.23) had no advantage over delayed PCI. At present, there are few studies specifically aimed at the timing of NSTEMI intervention. Although the VERDICT study also concluded that intervention therapy within 12 h could improve the prognosis, the research population was aimed at NSTE-ACS patients [17]. This study intended to conduct a subgroup analysis of NSTEMI within 24 h of intervention therapy, but the sample size was too small to be analyzed.

In addition, this study also concluded that for low-risk patients with NSTEMI with a GRACE score ≤ 108 points, early interventional therapy did not bring benefits to patients. This is inconsistent with the intervention within 24 h recommended by the guidelines, which may be related to the number of selected cases, and needs further study and demonstration. Of course, this study did not exclude critical patients such as mechanical complications, hemodynamics, and electrocardiographic instability, which may cause differences in research conclusions. For example, the randomized controlled trials such as the VERDICT study would exclude patients who are rapidly deteriorating due to medical ethics and other reasons [17].

Although European and American guidelines recommend that patients with NSTEMI should undergo coronary angiography within 24 h, people have insufficient attention to NSTEMI compared with STEMI, which leads to a common phenomenon of delayed NSTEMI treatment [21, 22]. One study reported that the proportion of patients receiving NSTEMI within 24 h of receiving PCI was only 36% and the proportion of delayed intervention treatment in China was even higher [25]. In this study, the proportion of patients receiving intervention treatment within 24 h was only 6.71%, which meant that the vast majority of patients failed to meet the requirements of the coronary angiography within 24 h of the guidelines. One of the reasons is the few clinical studies on the timing of NSTEMI intervention. There are many clinical studies on the relationship between the timing of intervention and the prognosis of patients with NSTE-ACS, but there are few studies on patients with NSTEMI and fewer related domestic studies. This study provides evidence for timing of intervention on patients with NSTEMI.

There are two main limitations of this study: first, this study is a real-world observational study, and the conclusions would require further randomized controlled trials to validate. Second, the cases of MACE and the number of interventions within 24 h in this study are small, which may affect the results of the survival analysis.

The results of this study show that the rate of intervention treatment of patients with NSTEMI within 24 h after admission in our center is comparatively low. In the future, we need to pay more attention to NSTEMI and improve the efforts of treatment through better procedures. In addition, no effective conclusions on interventional treatment strategies for patients with intermediate risk have been drawn and further exploration is needed.

## Figures and Tables

**Figure 1:** Kaplan-Meier survival curves of NSTEMI cohort 1-year and all-cause death, TLR, recurrent nonfatal AMI, severe HF requiring hospitalization, stroke, and MACE events (two ratios).

**Figure 2:** Forest chart of the subgroup analysis of the impact of the GRACE score and intervention time on MACE events.

**Figure 3:** Surface graph of the effect of interaction between GRACE score and intervention time on MACE events (applied the generalized additive model to fit GRACE score and intervention time on the surface of MACE events in patients with NSTEMI. The *z*-axis refers to the intervention treatment time grouping and GRACE score. The amount of partial effect of two indicators on survival time. It could be found from the figure that when the GRAEC score was low, the intervention time within >72 h had a higher survival time. Similarly, when the GRACE score was higher, the intervention time within 24 h had a higher survival time).

**Table 1:** Baseline characteristics.

Variables	Population (*N* = 1357)	GRACE scores ≤ 108 points (*N* = 413)	GRACE scores 109–140 points (*N* = 506)	GRACE scores > 140 points (*N* = 438)	*p*
Age (years)	64.72 ± 11.52	54.65 ± 9.69	65.86 ± 8.74	72.91 ± 8.42	≤0.001^∗∗^
Male, *N* (%)	945 (69.64)	328 (79.41)	369 (72.92)	248 (56.62)	≤0.001^∗∗^
Medical history, *N* (%)					
Hypertension	917 (67.58)	268 (64.89)	347 (68.57)	302 (68.95)	0.374
Diabetes mellitus	460 (33.90)	114 (27.60)	163 (32.21)	183 (41.78)	≤0.001^∗∗^
Stroke	312 (22.99)	55 (13.31)	119 (23.52)	138 (31.51)	≤0.001^∗∗^
Previous MI	250 (18.42)	54 (13.08)	92 (18.18)	104 (23.74)	≤0.001^∗∗^
Previous PCI	219 (16.14)	58 (14.04)	90 (17.79)	71 (16.21)	0.308
Previous CABG	73 (5.38)	13 (3.15)	27 (5.34)	33 (7.53)	0.018^∗^
Current smokers	790 (58.26)	279 (67.72)	303 (59.88)	208 (47.49)	≤0.001^∗∗^
Laboratory characteristics					
LVEF (%)	51.33 ± 9.86	55.11 ± 7.90	52.5 ± 8.79	46.41 ± 10.69	≤0.001^∗∗^
Serum creatinine (*μ*mol/L)	86.69 ± 30.58	76.30 ± 18.37	85.12 ± 27.04	98.09 ± 38.64	≤0.001^∗∗^
NT-proBNP (pg/mL)	2621.64 ± 4887.30	886.19 ± 2259.39	1643.33 ± 2881.87	5367.20 ± 6929.13	≤0.001^∗∗^
Hs-cTnT (ng/mL)	1.06 ± 1.47	0.68 ± 0.89	0.91 ± 1.17	1.59 ± 1.98	≤0.001^∗∗^
Treatment methods, *N* (%)					
Conservative treatment	472 (34.78)	99 (23.97)	158 (31.23)	215 (49.09)	≤0.001^∗∗^
PCI	770 (56.74)	286 (69.24)	30 1(59.48)	183 (41.78)	≤0.001^∗∗^
CABG	115 (8.47)	28 (6.78)	47 (9.28)	40 (9.13)	0.332
Time from admission to intervention therapy					
<24 h, *N* (%)	91 (6.71)	29 (7.02)	28 (5.53)	34 (7.76)	0.375
24–27 h, *N* (%)	110 (8.11)	48 (11.62)	42 (8.30)	20 (4.57)	0.001^∗∗^
>72 h, *N* (%)	509 (37.51)	189 (45.76)	208 (41.11)	112 (25.57)	≤0.001^∗∗^
Extent of coronary artery disease, *N* (%)					
0-Vessel	22 (2.05)	14 (3.77)	4 (0.96)	4 (1.41)	0.014^∗^
1-Vessel	177 (16.51)	83 (22.37)	69 (16.55)	25 (8.80)	≤0.001^∗∗^
2-Vessel	245 (22.85)	101 (27.22)	99 (23.74)	45 (15.85)	0.002^∗∗^
3-Vessel	623 (58.11)	172 (46.36)	242 (58.03)	209 (73.59)	≤0.001^∗∗^
LM disease, *N* (%)	165 (15.39)	27 (7.28)	62 (15.11)	75 (26.41)	≤0.001^∗∗^
≥1 vessel occlusion, *N* (%)	464 (34.19)	141 (34.14)	176 (34.78)	147 (33.56)	0.925

CABG: coronary artery bypass surgery; LVEF: left ventricular ejection fraction; LM: left main trunk.

**Table 2:** Comparison of general admissions of patients in the MACE group and non-MACE group.

Variables	MACE (*N* = 209)	Non-MACE (*N* = 1055)	*Z*/*χ*^2^	*p*
Age (years)	74 (67,80)	64 (56,71)	10.445	<0.0001^∗∗^
Male, *N* (%)	118 (56.46)	763 (72.32)	20.784	<0.0001^∗∗^
Hypertension, *N* (%)	150 (71.77)	707 (67.01)	1.807	0.179
Diabetes mellitus, *N* (%)	99 (47.37)	325 (30.80)	27.331	<0.0001^∗∗^
Stroke, *N* (%)	69 (33.01)	223 (21.13)	13.852	<0.0001^∗∗^
Current smokers, *N* (%)	96 (45.93)	641 (60.76)	15.772	<0.0001^∗∗^
Previous MI, *N* (%)	56(26.79)	185(17.53)	9.691	0.002∗
Previous PCI, *N* (%)	40 (19.14)	170 (16.11)	1.152	0.283
Previous CABG, *N* (%)	16 (7.66)	55 (5.21)	1.963	0.161
GRACE scores (points)				
≤108, *N* (%)	17 (8.13)	355 (33.65)	54.681	<0.0001^∗∗^
109–140, *N* (%)	57 (27.27)	426 (40.38)	12.692	<0.0001^∗∗^
>140, *N* (%)	135 (64.59)	274 (25.97)	118.88	<0.0001^∗∗^
LVEF (%)	55 (48,59)	45 (37,55)	−8.312	<0.0001^∗∗^
Serum creatinine(*μ*mol/L)	93.0 (75.0, 113.0)	78.0 (67.0, 94.0)	6.737	<0.0001^∗∗^
NT-proBNP (pg/mL)	3338.0 (1107.0, 8993.5)	753.7 (329.0, 1766.5)	11.995	<0.0001^∗∗^
Hs-cTnT (ng/mL)	0.9 (0.4, 2.1)	0.5 (0.2, 1.1)	6.143	<0.0001^∗∗^
Treatment methods				
Conservative treatment, *N* (%)	101 (48.33)	335 (31.75)	21.202	<0.0001^∗∗^
PCI, *N* (%)	87 (41.63)	623 (59.05)	21.515	<0.0001^∗∗^
CABG, *N* (%)	21 (10.05)	97 (9.19)	0.150	0.698
Extent of coronary artery disease, *N* (%)				
0-Vessel, *N* (%)	2 (0.96)	18 (1.71)	0.629	0.428
1-Vessel, *N* (%)	10 (4.78)	156 (14.78)	15.297	<0.0001^∗∗^
2-Vessel, *N* (%)	35 (16.75)	194 (18.39)	0.317	0.573
3-Vessel, *N* (%)	91 (43.54)	490 (46.45)	0.593	0.441
LM disease, *N* (%)	117 (55.98)	36 (3.41)	453.10	
≥1 vessel occlusion, *N* (%)	78 (37.32)	354 (33.55)	1.100	0.294

CABG: coronary artery bypass surgery; LVEF: left ventricular ejection fraction; LM: left main trunk.

**Table 3:** MACE event Cox multifactor regression analysis.

Variables	*β*	HR (95% CI)	*p*
Age (years)	0.034	1.035 (1.013-1.058)	0.002^∗^
Male, *N*	0.429	1.302 (0.874-1.963)	0.3100
Diabetes mellitus, *N*	0.110	0.935 (0.542-1.302)	0.0632
GRACE scores (points)			
≤108	Ref	Ref	Ref
109–140	0.369	1.477 (1.765-2.750)	0.2600
>140	1.248	3.482 (1.765-6.870)	<0.0001^∗∗^
Time from admission to treatment (hours)			
<24	Ref	Ref	Ref
24–72	0.673	1.966 (0.652,5.934)	0.2312
>72	1.612	4.989 (2.249,11.081)	<0.0001^∗∗^
Hs-cTnT (ng/mL)	0.143	1.153 (1.042,1.267)	0.0066^∗^
≥1 vessel occlusion	0.433	1.542 (1.038,2.273)	0.0301^∗^

## Data Availability

The data used to support the findings of this study are available from the corresponding author upon request.
